The article "Magnetic resonance imaging reconstruction algorithm under complex convolutional neural network in diagnosis and prognosis of cerebral infarction" was retracted in 2023. Reasons: duplicate publication; overlap with earlier publications; compromised peer review; unreliable results or conclusions.

# Magnetic resonance imaging reconstruction algorithm under complex convolutional neural network in diagnosis and prognosis of cerebral infarction

**DOI:** 10.1371/journal.pone.0251529

**Published:** 2021-05-17

**Authors:** Jie Dong, Shujun Zhao, Yun Meng, Yong Zhang, Suxiao Li

**Affiliations:** 1 School of Physics and Microelectronics, Zhengzhou University, Zhengzhou, P.R. China; 2 Department of Magnetic Resonance, The First Affiliated Hospital of Zhengzhou University, Zhengzhou, P.R. China; Ministry of Natural Resources North Sea Bureau, CHINA

## Abstract

This study was to explore the application value of magnetic resonance imaging (MRI) image reconstruction model based on complex convolutional neural network (CCNN) in the diagnosis and prognosis of cerebral infarction. Two image reconstruction methods, frequency domain reconstruction network (FDRN) and image domain reconstruction network (IDRN), were introduced based on the CCNN algorithm. In addition, they were integrated to form two new MRI image reconstruction models, namely D-FDRN and D-IDRN. The peak signal to noise ratio (PSNR) value and structural similarity index measure (SSIM) value of the image were compared and analyzed before and after the integration. The MRI images of patients with cerebral infarction in the dataset were undertaken as the data source, the average diffusion coefficient (DCavg) and apparent diffusion coefficient (ADC) values of different parts of the MRI image were measured, respectively. The correlation of the vein abnormality grading (VABG) to the infarct size and the degree of stenosis of the responsible vessel was analyzed in this study. The results showed that the PSNR and SSIM values of the MRI reconstructed image of the D-IDRN algorithm based on the CCNN algorithm in this study were higher than those of other algorithms. There was a positive correlation between the VABG and the infarct size (r = 0.48 and *P* = 0.002), and there was a positive correlation between the VABG the degree of stenosis of the responsible vessel (r = 0.58 and *P* < 0.0001). The ADC value of the central area of the infarct on the affected side was significantly greatly lower than that of the normal side (*P* < 0.01), and the DCavg value of the central area of the infarct was much lower in contrast to the normal side (*P* < 0.05). It indicated that an image reconstruction algorithm constructed in this study could improve the quality of MRI images. The ADC value and DCavg value changed in the infarct central area could be used as the basis for the diagnosis of cerebral infarction. If the vein was abnormal, the patient suffered from severe vascular stenosis, large infarction area, and poorer prognosis.

The article "Magnetic resonance imaging reconstruction algorithm under complex convolutional neural network in diagnosis and prognosis of cerebral infarction" was retracted in 2023. Reasons: duplicate publication; overlap with earlier publications; compromised peer review; unreliable results or conclusions.

## 1. Introduction

With the improvement of people’s living standards in recent years, the incidence of cerebral infarction has increased extremely, accounting for about 80% of all cerebrovascular diseases. Its high recurrence rate and disability rate have seriously affected the quality of life of patients [1]. Effective diagnosis and treatment of cerebral infarction at the early stage is of great significance to the occurrence of cerebral ischemic death and cerebral infarction complications. At present, imaging technology is mainly used to diagnose and treat patients with cerebral infarction. Compared with X-ray and computed tomography (CT) scanning technology, MRI has clearer scan images and relatively low ionizing radiation, so it is often used in the diagnosis and treatment of patients with cerebral infarction [2]. However, MRI technology still has some shortcomings. At present, MRI scan imaging takes a long time, so that the subject has to maintain the same posture for a long time during the detection process, which leads to the involuntary movement of the subject, and eventually causes motion artifacts, so as to bring greater impacts on the diagnosis and treatment of diseases [3]. Therefore, shortening the imaging time is a hotspot and focus in the field of MRI.

At present, the methods to speed up MRI imaging mainly include two ways: MRI hardware modification and reduction of K-space sampling data [4]. The latter method can speed up the MRI imaging through reconstruction algorithms, and it is featured with lower cost and higher imaging quality. With the development of deep learning technology in recent years, a theoretical foundation has been laid for reducing K-space sampling data and speeding up the MRI imaging. In 2016, Choi et al. (2016) [5] researchers applied convolutional neural network (CNN) to MRI image reconstruction for the first time, such end-to-end learning method not only speeded up the MRI reconstruction speed, but also improved the MRI image quality greatly. At the same time, researchers had combined the classic MRI reconstruction method based on compressed sensing with CNN to establish a Deep Cascaded CNN (DCCNN) reconstruction method, whose speed had been accelerated to a reliable degree in contrast to the traditional methods [6]. The MRI reconstruction method based on CCNN is improved on the basis of DCCNN. Although the CCNN algorithm improves the performance of MRI image reconstruction, it can’t effectively extract the complex-valued features.

To sum up, the incidence and disability rate of cerebral infarction were relatively high. MRI was often adopted to diagnose the cerebral infarction in clinical practice, but its imaging speed was slow relatively. The complex value K space was enriched based on the current CCNN reconstruction algorithm in this study. The MRI images of patients with cerebral infarction were undertaken as data to improve the performance of MRI reconstruction, and provide reference value for clinical diagnosis and prognosis of cerebral infarction lesions.

The article "Magnetic resonance imaging reconstruction algorithm under complex convolutional neural network in diagnosis and prognosis of cerebral infarction" was retracted in 2023. Reasons: duplicate publication; overlap with earlier publications; compromised peer review; unreliable results or conclusions.

## 2. Materials and methods

### 2.1 Experimental data

The MRI images of patients with cerebral infarction were derived from the public OpenfMRI data set and Figshare data set (https://doi.org/10.6084/m9.figshare.8851955). The collected data were from 72 volunteers, with 50 images from each volunteer. All MRI images were in the size of 256 × 256 and were complex MIR image data. The images included met the following criteria: the infarct was located in the cerebral hemisphere; the lesions were unilateral; the image quality could clearly show the lesion; and the data of the patients were complete. All personal information of patients in this database was anonymized using data encryption. The research procedure had been approved by the ethics committee of The First Affiliated Hospital of Zhengzhou University.

### 2.2 CCNN and its optimization

For a two-dimensional matrix *A*, the convolution operation of the matrix coordinates *(x*,*y)* could be expressed as Eq (1). In the equation, *K* was the convolution kernel; *S* was the convolution result, *m* referred to the number of neurons in the input layer, and *n* referred to the number of neurons in the output layer.

$$S\left(x,y\right)=\left(K*A\right)\left(x,y\right)=\sum_{m}\sum_{n}A\left(x-m,j-n\right)K\left(m,n\right)$$ (1)

*a* ϵ *C*^*N*^ *was* assumed as a vectorized MRI image with a complex pixel value, and the acceleration of this image had to restore the clarity of the MRI image *a* through the observed *b* ϵ *C*^*M*^ of the vectorized K-space, then the K-space observation *a* could be calculated with *b* = *F*_*μ*_*a*. Where, *F*_*N*_ was the sampled Fourier coding matrix, and *F*_*μ*_ ϵ *C*^*M×N*^ (*M* ≪ *N*). Then, the calculation method could be written as *F*_*μ*_ *=* *M*_*m*_*F*, where *M*_*m*_ referred to the sampling template, and *M*_*m*_ ϵ *C*^*M×N*^; *F* was the two-dimensional discrete Fourier transform, and *F* ϵ *C*^*N×N*^. For a general matrix image *a*_*f*_ in size of *M×N*, its *F* could be expressed as Eq (2) below:

$$F\left[k,l\right]=\frac{1}{\sqrt{MN}}\sum_{n=0}^{N-1}\sum_{m=0}^{M-1}a_{f}\left(m,n\right)e^{-y2\pi \left(\frac{mk}{M}+\frac{nl}{N}\right)},\left(0\leq m,k\leq M-1,0\leq n,1\leq N-1\right)$$ (2)

When only the K-space observation *b* was obtained, the above algorithm was difficult to solve for *a*, and it was necessary to add constraints to *a* to solve the problem, which could be expressed as follows:

$$\underset{a}{\min}\beta \left(a\right)+\kappa {\left\|b-F_{\mu }a\right\|}_{2}^{2}$$ (3)

In the above equation, *β* was the constraint term imposed on *a*; and *k* was the regularization parameter. Then, the constraint based on the deep learning model could be expressed as $\underset{a}{\min}{\left\|a-f\left(a|\theta \right)\right\|}_{2}^{2}+\kappa {\left\|F_{\mu }a-b\right\|}_{2}^{2}$, where *f* was the deep learning model.

The article "Magnetic resonance imaging reconstruction algorithm under complex convolutional neural network in diagnosis and prognosis of cerebral infarction" was retracted in 2023. Reasons: duplicate publication; overlap with earlier publications; compromised peer review; unreliable results or conclusions.

In order to obtain a clear MRI mapping image, the data fidelity item was combined with the CNN. The known information was mainly obtained from the reconstruction result of K-space observation *b*, which could be expressed as Eq (4) below:

$$a_{rec}=f\left(a_{\mu }|\theta ,\Omega \right)$$ (4)

In the above equation, Ω referred to index from K-space observation *y*, *θ* represented the parameter of the CNN model, and *a*_*rec*_ was the prediction result of the CNN model. A training pair (*a*_*μ*_,*a*_*g*_) was formed by the MRI image *a*_*μ*_ with artifacts and a clear MRI image *a*_*g*_, then the Eq (5) could be adopted for training. Where, *ε* was the loss function used to train the network.

$$M\left(\theta \right)=\sum \varepsilon \left(a_{\mu },a_{g}\right)$$ (5)

In order to ensure the fidelity term could be integrated in the network model, the network model parameter *θ* was assumed as a fixed value, then the final K-space result output after the fidelity term was added to the network model could be expressed as follows:

$${\hat{a}}_{recon}\left(k\right)=\{\begin{array}{cc} {\hat{a}}_{rec}\left(k\right) & \\ \frac{{\hat{a}}_{rec}\left(k\right)+\kappa {\hat{a}}_{\mu }\left(k\right)}{1+\kappa } & \begin{array}{c} k\notin \Omega \\ k\in \Omega \end{array} \end{array}$$

$$=\{\begin{array}{cc} {\hat{a}}_{rec}\left(k\right) & \\ \frac{{\hat{a}}_{rec}\left(k\right)+\kappa b}{1+\kappa } & \begin{array}{c} k\notin \Omega \\ k\in \Omega \end{array} \end{array}$$ (6)

In the above equation, the index *k* was the closed-form solution in K-space, *κ* was the constant, and ${\hat{a}}_{rec}$ was the Fourier transform of the network model output *a*_*rec*_. ${\hat{a}}_{\mu }$ was the Fourier transform of the network model input *a*_*μ*_, which referred to the K-space observation *b*. ${\hat{a}}_{recon}$ was the final output K-space result after the fidelity term was added to the network model, which was performed with the Fourier transform to obtain the MRI image finally outputted by the network model after the fidelity term was added. *k* ϵ Ω indicated the observed value by transforming the predicted MRI image into the K-space.

The article "Magnetic resonance imaging reconstruction algorithm under complex convolutional neural network in diagnosis and prognosis of cerebral infarction" was retracted in 2023. Reasons: duplicate publication; overlap with earlier publications; compromised peer review; unreliable results or conclusions.

For the K-space matrix ${\hat{a}}_{in}=Fa_{in}$ corresponding to the two-dimensional matrix *a*_*in*_, its final output of the K-space result could be expressed as $f_{kc}\left({\hat{a}}_{in},{\hat{a}}_{\mu s},\kappa \right)=\forall {\hat{a}}_{in}+\frac{\kappa }{1+\kappa }{\hat{a}}_{\mu s}$. Where, ${\hat{a}}_{\mu s}$ was the Fourier transform of *a*_*μs*_, *a*_*μs*_ was the matrix form of the MRI image *a*_*μ*_ with artifacts inputted by the network. In addition, ∀ was the diagonal matrix, and could be calculated with $\forall_{kk}=\left\{ \begin{array}{ll} 1 & \\ \frac{1}{1\text{+}\kappa } & \begin{array}{l} k\notin \Omega \\ k\in \Omega \end{array} \end{array}\right.$. The corrected K-space value was transformed into the image domain to obtain the forward transfer process of the K-space correction layer. Then, the calculation method for the result of the forward transfer was given as follows:

$$f_{LP}\left(a_{in},{\hat{a}}_{in},\kappa \right)=F^{-1}\forall Fa_{in}+F^{-1}{\hat{a}}_{in}\frac{\kappa }{\left(1+\kappa \right)}$$ (7)

The back propagation gradient was calculated further. The effect of the two-dimensional discrete Fourier transform matrix *F* was regarded as a linear transformation process of *a*_*in*_, then the derivative result of *a*_*in*_ by *f*_*LP*_ was $\frac{\partial f_{LP}}{\partial a_{in}}=F^{-1}\forall F$.

The original K-space data was a complex number data, which could be expressed as *y* = *c* + *di*. Where, *c* was the real number of the real part; and *d* was the real number of the imaginary part. When the weight *W* = *C* + *Di* was inputted, the complex convolution algorithm could be written as Eq (8) below:

W*y=(C*c−D*d)+i(D*c−C*d) (8)

After complex convolution, the corresponding complex-valued feature map was obtained. The real and imaginary part of the complex-valued feature map could be expressed as follows:

$$\left[\begin{array}{l} \text{Re}\left(W*y\right)\\ \text{Im}\left(W*y\right) \end{array}\right]=\left[\begin{array}{l} C-D\\ D_{}{}_{{{}_{}}_{}}C \end{array}\right]*\left[\begin{array}{l} c\\ d \end{array}\right]$$ (9)

Thus, the real and imaginary part of the complex-valued feature map obtained after complex convolution was Re(*W* * *y*) = *C* * *c*–*D* * *d* and Im(*W* * *y*) = *D* * *c* + *C* * *d*, respectively. For N feature maps, the first *N*/2 feature maps were the real part, and the latter *N*/2 feature maps were the imaginary part. The number of output feature maps in the next layer was *M*. If the weight size was equal to *m* × *m*, then the size of both the real part and the imaginary part of the weight was *m* × *m*, and then the amount of parameters to learn from the current layer to the next layer was $\frac{N\times M\times m\times m}{2}$.

The article "Magnetic resonance imaging reconstruction algorithm under complex convolutional neural network in diagnosis and prognosis of cerebral infarction" was retracted in 2023. Reasons: duplicate publication; overlap with earlier publications; compromised peer review; unreliable results or conclusions.

### 2.3 Establishment of reconstructed MRI image based on CCNN

The image reconstruction process based on CCNN was shown in Fig 1. For MRI images with artifacts, the network MRI image was inputted after calculation by CCNN calculation method, and then was further processed by the K-space correction layer. The processed image was returned to the CCNN calculation method and the K-space correction layer for further processing. Such operations were repeated for many times to increase the definition of the MRI image, and the obtained MRI image with higher definition was reconstructed through the MRI reconstruction image to finally obtain the MRI reconstruction image.

**Fig 1:** Calculation process of CCNN.

In order to further increase the quality and calculation speed of the MRI image, a dual-domain reconstruction model was adopted to reconstruct the MRI image after the K-space correction processing under CCNN operation. As shown in Fig 2, it mainly included the K-space reconstruction model (FDRN) and IDRN, which were merged. When the FDRN and IDRN methods were adopted for separate reconstruction, each basic reconstruction module could interact with information. The upper branch image domain reconstruction branch was named D-IDRN, and the lower K-space reconstruction branch was named D-FDRN.

**Fig 2:** A dual-domain reconstruction model of MRI image.

### 2.4 Quality evaluation indicators for reconstructed MRI image based on CCNN

The quality of the reconstructed MRI image was evaluated with two major indicators: PSNR and SSEM. The higher the PSNR value, the better the quality of the reconstructed MR image. The calculation method of PSNR was defined as $PSNR=10\text{lg}\left[\frac{{\left(2^{n}-1\right)}^{n}}{MSE}\right]$. Where, *n* was the number of bits per pixel; *MSE* referred to the mean square error between the two images and could be calculated with $MSE=\frac{1}{H\times W}{\sum_{i=1}^{H}\sum_{j=1}^{W}\left[X\left(i,j\right)-Y\left(i,j\right)\right]}^{2}$. Where, *H* and W referred to the height and width of the MRI image to be measured, respectively, *X* was the reconstructed MRI image, and *Y* was the original MRI image.

SSIM modelled the distortion of the reconstructed MRI image as a combination of three different attributes, which were contrast, brightness, and structural information. The SSIM could be calculated with $SSIM\left(X,Y\right)=\frac{\left(2\mu_{x}\mu_{\gamma }+e_{1}\right)\left(2\sigma_{x\gamma }+e_{2}\right)}{\left(\mu^{2}{}_{x}+\mu^{2}{}_{\gamma }+e_{1}\right)\left(\sigma^{2}{}_{x}+\sigma^{2}{}_{\gamma }+e_{2}\right)}$, where *μ*_*x*_ and *μ*_*γ*_ were the mean values of *X* and *Y*, respectively, *σ*^2^_*x*_ and *σ*^2^_*γ*_ were the variances of *X* and *Y*, respectively, and *e*_1_ and *e*_2_ were constants that maintained the stability.

The article "Magnetic resonance imaging reconstruction algorithm under complex convolutional neural network in diagnosis and prognosis of cerebral infarction" was retracted in 2023. Reasons: duplicate publication; overlap with earlier publications; compromised peer review; unreliable results or conclusions.

### 2.5 Measurement of infarct size and grading of stenosis degree of the responsible vessel

The largest layer of the lesion on the MRI image was selected and the edge of the lesion was outlined to obtain the infarct size. For multiple infarcted lesions, the area of each lesion should be calculated separately, and then summed to obtain the total area. The infarct size was classified according to the Adams standard: large infarct lesion: infarct area > 5 cm; middle infarct lesion: 3 cm < infarct area < 5 cm; and small infarct lesion: infarct area < 3 cm [7].

According to the research results of Li et al. (2015) [8], the degree of MRI vascular stenosis was divided into 4 grades: grade 0 referred to the normal blood vessels; grade 1 indicated mild stenosis with a stenosis rate ≤ 50%; grade 2 suggested moderate and severe stenosis with a stenosis rate > 50%; and grade 3 suggested occlusion without development of distal blood vessels.

### 2.6 Evaluation basis and prognosis evaluation method of MRI images for cerebral infarction

The distributions of cerebral veins in the brain hemispheres in the affected and health side on the MRI image were compared, and it could be defined as abnormality if the number of veins was increased or the vessel wall was thickened [9]. Cerebral venous abnormalities mainly included: grade 0 (no visible changes in the two measured cerebral veins), grade 1 (the cerebral vein of the diseased side was slightly increased or thicker than the healthy side); and grade 2 (the cerebral vein on the affected side was obviously increased and thicker than that on the healthy side) [10].

The DCavg value and ADC value of MRI images were measured, respectively. In addition, they were compared in the semi-oval center, lenticular nucleus, the posterior horn of the lateral ventricle, the forelimb of the internal capsule, the hind limbs, the knee and the infarct central area, the marginal area, and the normal area around the focus.

### 2.7 Statistical methods

The test data was processed using SPSS19.0 statistical software. The measurement data was expressed as mean ± standard deviation ($\bar{x}$ ± s), and count data was indicted by a percentage (%). The χ^2^ test was adopted. The DCavg and ADC values in the infarct central area, the marginal area, and the normal area around the focus were analyzed using ANOVA. *P* < 0.05 indicated that the difference was statistically significant.

## 3. Results

### 3.1 Quality analysis on image of the reconstruction algorithm based on CCNN

The PSNR and SSIM values without FDRN, IDRN, D-IDRN, and D-FDRN were compared and analyzed, and the results were shown in Fig 3. It illustrated that the D-IDRN and D-FDRN images after fusion of FDRN and IDRN showed higher PSNR and SSIM value than those before the integration. In addition, the PSNR and SSIM value of the D-IDRN image were both higher than those of the D-FDRN image under different number of reconstruction modules.

The article "Magnetic resonance imaging reconstruction algorithm under complex convolutional neural network in diagnosis and prognosis of cerebral infarction" was retracted in 2023. Reasons: duplicate publication; overlap with earlier publications; compromised peer review; unreliable results or conclusions.

**Fig 3:** Quality analysis on reconstructed images under different models. Note: Fig 3A and 3B illustrated the comparisons of PSNR and SSIM of the reconstructed image under different models, respectively.

Then, the PSNR and SSIM values of the reconstructed images of different models were analyzed and compared further under different sampling rates. The results shown in Fig 4 illustrated that the PSNR and SSIM values of D-IDRN were higher than those of other reconstructed model.

**Fig 4:** Quality analysis on reconstructed images under different sampling rates. Note: Fig 4A and 4B illustrated the comparisons of PSNR and SSIM of the reconstructed image under different sampling rates, respectively.

### 3.2 MRI image characteristics of cerebral infarction

The MRI image characteristics of patients with cerebral infarction were shown in Fig 5. The MRI image had a high signal infarct in the apical junction area (Fig 5A), and the lesion had a low signal in the DWI image (Fig 5B). The branches of the distal middle cerebral artery were sparse (Fig 5C); the veins around the infarct were slightly increased and thickened (Fig 5D); and the posterior artery branches were obviously thicker and longer than those of the contralateral side (Fig 5E).

**Fig 5:** MRI image characteristics of cerebral infarction. Note: Fig 5A, 5C–5E referred to the MRI images of lesion, cerebral artery, degree of vessel stenosis, and vessel branches, respectively; and 5B showed a DWI image of lesion.

### 3.3 Correlation of VABG to infarct size and degree of stenosis of the responsible vessel

The correlation between VABG and infarct size was analyzed based on the detection results of VABG and infarct size of MRI images, and the results were shown in Fig 6. It revealed that the patient’s VABG became more severe as the infarct size increased. Therefore, there was a positive correlation between VABG and infarct size (r = 0.48, *P* = 0.002).

**Fig 6:** Correlation between VABG and infarct size.

According to the results of VABG and the degree of stenosis of the responsible vessel of the MRI image, the correlation between them was analyzed. As shown in Fig 7, there was a positive correlation between VABG and the degree of stenosis of the responsible vessel (r = 0.58, *P* < 0.0001).

The article "Magnetic resonance imaging reconstruction algorithm under complex convolutional neural network in diagnosis and prognosis of cerebral infarction" was retracted in 2023. Reasons: duplicate publication; overlap with earlier publications; compromised peer review; unreliable results or conclusions.

**Fig 7:** Correlation between VABG and degree of stenosis of the responsible vessel.

### 3.4 Comparison on ADC and DCavg of different brain parts in the affected and normal side

The ADC values of different brain parts of the affected side and the normal side in the MRI image were compared, and the results were shown in Fig 8. It disclosed that there was no observable difference among the ADC values in semi-oval center, the posterior horn of the lateral ventricle, the forelimb of the internal capsule, knee of internal capsule, the hind limbs of internal capsule, lenticular nucleus, the brain stem, the marginal area of infarct focus, and the normal area around the focus in both sides (*P* > 0.05); while the ADC value in infarct central area in the affected side was dramatically lower than that in the normal side (*P* < 0.01).

**Fig 8:** Comparison on ADC values different brain parts in the affected and normal side. A–J referred to the semi-oval center, the posterior horn of the lateral ventricle, the forelimb of the internal capsule, knee of internal capsule, the hind limbs of internal capsule, lenticular nucleus, the brain stem, the infarct central area, the marginal area of infarct focus, and the normal area around the focus, respectively. (** indicated the difference was huge in contrast to the affected side (*P* < 0.01)).

The DCavg values of different brain parts of the affected side and the normal side in the MRI image were compared, and the results were shown in Fig 9. It disclosed that there was no observable difference among the DCavg values in semi-oval center, the posterior horn of the lateral ventricle, the forelimb of the internal capsule, knee of internal capsule, the hind limbs of internal capsule, lenticular nucleus, the brain stem, the marginal area of infarct focus, and the normal area around the focus in both sides (*P* > 0.05); while the DCavg value in infarct central area in the affected side was dramatically lower than that in the normal side (*P* < 0.05).

**Fig 9:** Comparison on DCavg values different brain parts in the affected and normal side. A–J referred to the semi-oval center, the posterior horn of the lateral ventricle, the forelimb of the internal capsule, knee of internal capsule, the hind limbs of internal capsule, lenticular nucleus, the brain stem, the infarct central area, the marginal area of infarct focus, and the normal area around the focus, respectively. (** indicated the difference was huge in contrast to the affected side (*P* < 0.01)).

## 4. Discussion

The CCNN network is one of the most successful MRI reconstruction models [11]. When the complex MRI data was processed, the difference between the complex residual module based on complex convolution and the real residual module based on real convolution was that the calculation process of each layer of the network was different and the resulting feature map arrangements were different [12]. To obtain high-quality reconstructed images after integration of multiple models, it was necessary to combine the common points of these fusion algorithms to improve the algorithm and the image quality [13]. The MRI images were reconstructed based on the CCNN algorithm in this study. In the reconstruction process, two image reconstruction methods (FDRN and IDRN) were used, and both methods had complex residual modules and K-space correction layers in the reconstruction process, which provided basis for information interaction and integration of them. The quality of the reconstructed images of the single-domain reconstruction model FDRN and IDRN and the double-domain reconstruction model D-FDRN and D-IDRN was evaluated comprehensively. It was found that the PSNR and SSIM value of the D-IDRN reconstruction algorithm under different reconstruction modules and sampling rates were higher than those of other models. The average PSNR value of the D-IDRN algorithm under different reconstruction modules and sampling rates was 7.04dB and 4.15dB larger than that of the FDRN algorithm, respectively, indicating that the D-IDRN dual-domain reconstruction model established in this study could extremely improve the quality of MRI images.

The article "Magnetic resonance imaging reconstruction algorithm under complex convolutional neural network in diagnosis and prognosis of cerebral infarction" was retracted in 2023. Reasons: duplicate publication; overlap with earlier publications; compromised peer review; unreliable results or conclusions.

In the imaging examination of cerebral infarction, it is of important research significance to provide reference information for clinical treatment plan and prognosis through the image at the time of diagnosis. After the occurrence of cerebral infarction, an ischemic penumbra appears around the infarct [14]. If effective treatment is implemented in time, the patient’s “ischemic penumbra” can be relieved to the greatest extent, otherwise the infarct can be expanded further. Therefore, measuring and judging the local cerebral blood flow state and the viability of brain tissue in patients with cerebral infarction if of critical significance to accurately assess the condition of patients with clinical practice. The results of this study found that there was a positive correlation between VABG and infarct size (r = 0.48, *P* = 0.002). It might be because that the increased infarct size could cause an increase in the degree of cerebral ischemia, which in turn increased the deoxyhemoglobin content in the local venules, and eventually led to an increase in veins, so that the VABG was more obvious [15]. Wang et al. (2018) [16] showed that the larger the infarct size, the more obvious the perifocal VABG, which was similar to that of this study. Besides, there was a positive correlation between VABG and the degree of vessel stenosis (r = 0.58, *P* < 0.0001), indicating that the more severe the vessel stenosis, the more observable the VABG [17]. The reason might be that when the cerebral ischemia and hypoxia occurred in patients with cerebral infarction, the fractional venous oxygen uptake around the lesion increased compensatively. Once the patient’s responsible vessel was severely stenosis or occlusion, the degree of cerebral ischemia and hypoxia could increase extremely, leading to visible thickening and increasing of the veins around the lesion [18].

The article "Magnetic resonance imaging reconstruction algorithm under complex convolutional neural network in diagnosis and prognosis of cerebral infarction" was retracted in 2023. Reasons: duplicate publication; overlap with earlier publications; compromised peer review; unreliable results or conclusions.

The results of this study suggested that the ADC value of the infarct central area on the affected side of cerebral infarction patients was much lower than that of the normal side (*P* < 0.01). Animal research results show that [19], arterial embolism could cause a visible decrease in ADC value in the center of the lesion within 27 minutes. In addition, studies had pointed out [20] that the ADC value of the infarct central area in patients with cerebral infarction showed a rapid decline after an infarction, which was mainly caused by the diffusion limitation caused by edema [21]. The results of this study showed that the DCavg value of the infarct central area on the affected side was greatly lower than that on the normal side (*P* < 0.05). In the early stage of edema, there are changes in cell swelling, which reduces the gap between cells, in turn leads to an observable decrease in the DCavg value [22].

## 5. Conclusion

A MRI image reconstruction model was constructed based on CCNN, and the changes in image quality of the model were analyzed in this study. In addition, the reconstructed model was applied to the diagnosis and prognosis of cerebral infarction lesions. It was found that the PSNR and SSIM values of the image reconstructed by the new D-IDRN algorithm based on the CCNN algorithm were higher than those of other models; VABG was closely positively correlated to the infarct size and the degree of vessel stenosis; and the ADC value and DCavg value of the affected side were lower than those in the normal side. However, there were still some shortcomings in the research of this study. Because the MRI data of cerebral infarction included in this study was derived from a data set, its detection methods might be different, causing the results biased. In future work, it will collect the relevant data of patients with cerebral infarction for further test. In summary, an image reconstruction algorithm that could improve the quality of MRI images was established in this study; the ADC value and DCavg value changes in the infarct central area could be undertaken as the basis for the diagnosis of cerebral infarction. In addition, if the vein was abnormal, the patient suffered severe vessel stenosis, and the larger the size, the worse the prognosis. It provided a reference basis for the diagnosis and prognosis of clinical cerebral infarction.

The article "Magnetic resonance imaging reconstruction algorithm under complex convolutional neural network in diagnosis and prognosis of cerebral infarction" was retracted in 2023. Reasons: duplicate publication; overlap with earlier publications; compromised peer review; unreliable results or conclusions.

## Supporting information

S1 Data (ZIP)
